RETRACTED

# A new inducible transgenic mouse model for C9orf72-associated GGGGCC repeat expansion supports a gain-of-function mechanism in C9orf72-associated ALS and FTD

**DOI:** 10.1186/s40478-014-0166-y

**Published:** 2014-12-13

**Authors:** Renate K Hukema, Fréderike W Riemslagh, Shamiram Melhem, Herma C van der Linde, Lies-Anne WFM Severijnen, Dieter Edbauer, Alex Maas, Nicolas Charlet-Berguerand, Rob Willemsen, John C van Swieten

**Affiliations:** 1 Department of Clinical Genetics, Erasmus Medical Center, 3015 CE Rotterdam, The Netherlands; 2 Department of Neurology, Erasmus Medical Center, 3015 CE Rotterdam, The Netherlands; 3 German Center for Neurodegenerative Diseases, 81337 Munich, Germany; 4 Department of Cell Biology, Erasmus Medical Center, 3015 CE Rotterdam, The Netherlands; 5 Department of Neurobiology and Genetics, IGBMC, INSERM U964, CNRS UMR7104, University of Strasbourg, Illkirch, France; 6 Department of Neurology, Neuroscience Campus Amsterdam, 1007 MB Amsterdam, The Netherlands; 7 PO Box 2040, , 3000 CA Rotterdam, The Netherlands

**Keywords:** C9orf72, GGGGCC repeat, ALS, FTD, Inducible mouse model, RNA gain-of-function

Frontotemporal dementia (FTD) and amyotrophic lateral sclerosis (ALS) are two neurodegenerative disorders that share clinical, genetic and pathological overlap. In 2011, a hexanucleotide repeat (GGGGCC) expansion in the ‘chromosome 9 open reading frame 72’ (C9orf72) gene was identified as a cause of FTD and ALS [1,2]. This mutation has proven to be the most common genetic defect in the neurodegenerative field, especially in FTD and ALS [3]. Patients harboring the C9orf72 repeat expansion can develop FTD, ALS or both and are therefore associated with wide clinical diversity [4]. There have been multiple hypotheses about the underlying mechanisms by which the repeat expansion leads to neuropathology, including loss-of-function caused by haploinsufficiency of the endogenous C9orf72 protein product or gain-of-function induced by either RNA or protein toxicity. Either free RNA molecules containing the repeat expansion or RNA foci that sequester proteins could be toxic for cells. Alternatively, a pathogenic mechanism has been proposed for the production of toxic dipeptide repeat proteins (DPR) by repeat-associated non-AUG translation (RAN) of the repeat [5,6]. Interestingly, to differentiate between repeat “RNA-only” and DPR protein toxicity fruit fly models carrying a range of pure and RNA-only repeats have been generated. These studies demonstrated that the major toxic species were the DPR proteins [7].

Here we report on an “RNA-only” gain-of-function mouse model. To study the intrinsic effect of the repeat without assessing its effect on the C9orf72 gene, we created a spatially and temporally inducible transgenic mouse model. This mouse model has a repeat size of 80 GGGGCC-repeats, without human flanking regions, which may affect repeat translation. This repeat was cloned in the 5′ UTR of a GFP reporter gene and controlled by a tetracycline responsive element (TRE) promoter (Figure 1A). To enable expression of the TRE-construct we created bigenic mice that possess both the TRE-construct and the tetracycline-responsive transcriptional activator (rtTA) under a general heterogeneous nuclear ribonucleoprotein (hnRNP) promoter [8]. Expression of the repeat was turned on after weaning by adding doxycycline (dox) to the drinking water. Expression of the repeat construct can be stopped at any time by withdrawal of dox, allowing for reversibility studies (Figure 1A; more information about the creation of the model can be found in Additional file 1). After generation of transgenic mice, the repeat size remained stable for multiple generations (data not shown). GFP expression was seen in bigenic mice as soon as 4 days after dox treatment started and remained stable over time (assessed by western blot of liver homogenates, data not shown). Next to liver, multiple other tissues showed GFP expression including lung, kidney and brain; with most prominent expression in the striatum (Figure 1B) and the cuneate nucleus in the brainstem.

RETRACTED

**Figure 1:** **Expression of 80GGGGCC-repeats leads to the formation of ubiquitin-positive inclusions in mouse brain. A)** Schematic of the model used to create the inducible mice. Simultaneous expression of rtTA and doxycycline treatment are needed to drive expression of the TRE-80GGGGCC-eGFP construct. PCR for determining repeat size in three transgenic mice containing the repeat construct. **B)** GFP expression in the striatum of bigenic mice after 12 weeks dox treatment. **C)** Intranuclear (arrows) and neuropil (arrowheads) ubiquitin-positive inclusionsin the striatum of bigenic mice after 12 weeks dox treatment.

Both ubiquitin-positive, TDP-43-positive and TDP-43 negative neuronal and cytoplasmic inclusions are pathological hallmarks in post mortem brain tissue from C9orf72 FTD and ALS patients. We used the presence of inclusions as a readout for the effect of expression of the repeat in our “RNA-only” gain-of-function ALS/FTD model [9,10]. We found ubiquitin-positive inclusions in those brain regions that express high levels of GFP, including the striatum (Figure 1C) and the cuneate nucleus of bigenic mice after twelve weeks of dox treatment (n = 7 mice per group). Inclusions were found in the nuclei and the neuropil in striatum and mainly in the nuclei in the cuneate nucleus. The presence of ubiquitin-positive inclusions in our mouse model is a shared phenomenon with non-C9orf72 mouse models of ALS and FTD [11,12]. We did not observe any TDP-43 positive nor p409/410 TDP-43 positive inclusions in our mouse model after twelve weeks of dox treatment, despite the positive staining in a C9orf72 patient hippocampus control (data not shown). TDP-43 inclusions might only appear after prolonged expression of the repeat or additional genetic or environmental factors might be needed to drive TDP-43 dysfunction. Importantly, TDP-43 function could also be affected without the presence of TDP-43 positive aggregates [13]. The absence of DPR pathology was assessed with a poly-GA antibody [6]. We could not detect poly-GA aggregation in brain tissue from bigenic mice, but only revealed GA-positive inclusions in C9orf72 patient hippocampus control material illustrating lack of DPR pathology in this mouse model (Figure 2). The mice did not develop any obvious behavioral phenotype and showed no cell loss. The neurotoxic effect of the C9orf72 hexarepeat expansion has been suggested by both RNA- and protein-mediated pathology [7]. Due to lack of DPR pathology, this mouse is a good model to investigate whether toxicity can be driven by the repeat RNA only. Future studies focusing on molecular changes and behavior deficits in our mouse model can provide additional insight in disease progression, reversibility and create options for therapeutic intervention. In conclusion, we demonstrate that solely expression of the GGGGCC repeat outside the C9orf72 context results in ubiquitin-positive inclusions, which is a pathological hallmark in postmortem brain from ALS and FTD patients. Our data on this first C9orf72 mouse model argues in favor for a gain-of-function pathological mechanism in C9orf72 associated ALS and FTD.

RETRACTED

**Figure 2:** **Absence of DPR pathology in brain of 80GGGGCC RNA expressing mouse. A)** GA positive inclusions in the hippocampus of C9orf72FTD patient. **B)** the striatum of bigenic mice treated with dox for 12 weeks shows no GA positive inclusions.

All animal experiments were conducted with the permission of the local animal welfare committee (DEC). Experiments on human brain material were done under informed consent and approved by the Medical Ethical Test Committee (METC). Human paraffin embedded brain material was provided by the Dutch brain bank (Nederlandse Hersenbank NHB).

## Additional file

Additional file 1: **Supplementary material and methods.**

## Abbreviations

ALS: Amyotrophic lateral sclerosis
FTD: Frontotemporal dementia
C9orf72: Chromosome 9 open reading frame 72
DPR: Dipeptide repeat proteins
RAN: Repeat-associated non-AUG
TRE: Tetracycline responsive element
rtTA: Tetracycline-responsive transcriptional activator
hnRNP: Heterogeneous nuclear ribonucleoprotein
dox: Doxycycline
